The article "Progression Rate of Visual Function and Affecting Factors at Different Stages of Retinitis Pigmentosa" was published in 2022. Journal: Biomed Res Int.

# Progression Rate of Visual Function and Affecting Factors at Different Stages of Retinitis Pigmentosa

**DOI:** 10.1155/2022/7204954

**Published:** 2022-07-14

**Authors:** Nana Ito, Gen Miura, Yuki Shiko, Yohei Kawasaki, Takayuki Baba, Shuichi Yamamoto

**Affiliations:** ^1^Department of Ophthalmology and Visual Science, Chiba University Graduate School of Medicine, Chiba, Japan; ^2^Biostatistics Section, Clinical Research Centre, Chiba University Hospital, Chiba, Japan; ^3^Faculty of Nursing, Japanese Red Cross College of Nursing, Tokyo, Japan

## Abstract

We reviewed medical records of 121 patients/235 eyes of typical retinitis pigmentosa (RP) patients who could be followed up for at least 5 years with the aim of investigating the long-term course of visual function progression at each RP stage and appropriate assessment methods. Patients were classified into three groups: mild RP (baseline mean deviation (MD) ≥ −5), moderate RP (−25 < baseline MD < −5), and late RP (baseline MD ≤ −25). Linear mixed-effect models were used to follow MD, the average retinal sensitivity of the central four points of the Humphrey field analyzer 10-2 program (S4), and visual acuity (VA) with increasing time. The associations among factors (baseline MD group, sex, hereditary form) and the interaction between each factor and time were also investigated. The mean reduction of the MD, S4, and VA for all patients was -0.37 dB/year, -0.25 dB/year, and 0.018/year, respectively. The moderate RP group had a faster progression than other groups in MD (-0.43 dB/year, *p* < 0.05). The moderate (-0.31 dB/year, *p* = 0.01) and late RP groups (-0.25 dB/year, *p* < 0.01) had faster progression than the mild RP group in S4. The late RP group had faster progression in VA than the other groups (0.03/year, *p* < 0.05). Females had a slower progression of the S4 (-0.15 dB/year, *p* = 0.02) and VA (0.01/year, *p* < 0.001) than males. The autosomal dominant group had a slower progression than the sporadic group in MD (-0.22 dB/year, *p* = 0.02); the autosomal dominant and autosomal recessive groups had a slower VA decline than the sporadic group (0.01/year, *p* = 0.03; 0.01/year, *p* = 0.04). Because the progression rates of VA and visual field test differed as per the RP stage, S4 and VA can also be useful assessment methods depending on the stage. Inheritance form and sex may affect the progression rate.

## 1. Introduction

Retinitis pigmentosa (RP) is a genetic retinal dystrophy that results from the progressive loss of photoreceptor cells. The characteristic signs and symptoms of RP include impaired night vision, a gradual loss of the visual field, and eventual decline in visual acuity (VA) [1]. Owing to the progressive nature of RP, the development of therapeutic interventions to slow down the progression of the disease is required. The efficacy of therapeutic treatment options, including supplements (for example, vitamin A [2, 3], docosahexaenoic acid [4], brimonidine [5], lutein [6], and nilvadipine [7]) and oxygen therapy [8], is not conclusive. Several therapeutic options have been studied, including gene therapy [9], transplantation [10], optogenetic therapy [11], retinal prosthesis [12], and electrical stimulation [13]. To predict the prognosis of RP and assess the safety and efficacy of the new treatments, the natural course of RP should be known, and appropriate parameters must be established. Previous studies have reported the progression of visual field defects in RP patients by analyzing the change in the area of an isopter using Goldmann kinetic perimetry [14–16]. However, it is difficult to quantitatively evaluate the central visual field defect progression using Goldmann kinetic perimetry [17].

Previous studies suggested that the Humphrey field analyzer (HFA) is a suitable method to detect visual field loss [14, 16]. Several studies have investigated the progression of defects in the HFA10-2 program and indicated that the mean deviation (MD) value and central 4 points in the HFA10-2 perimetry were reasonable parameters to monitor the progression of RP [18–21]. However, the number of participating patients was few in those studies, and the natural course of progression in visual function was not conclusive.

Although some studies implied that the logarithm of the minimum angle of resolution (logMAR) VA is less suitable than perimetric parameters [19, 22], the perceived difficulty in performing common daily tasks was more strongly related to the level of VA than the residual visual field area for patients with RP [23]. Therefore, monitoring VA in addition to perimetric sensitivity is important. So far, few studies have examined the long-term natural course of RP using the HFA10-2 or VA tests, and whether the rate of progression varies with the stage of the disease is not clear. Moreover, several reports have investigated the difference in the rate of disease progression in terms of hereditary, form, and sex [24–26], and a few studies have indicated that progestin therapy appears to control the course of RP [27–29]. Thus, the aim of this study was to investigate the long-term course of the progression of visual function in RP patients and assess the difference in the rate of progression of visual function with the different stages of RP. We retrospectively analyzed the annual progression of visual function in RP patients using the results of the HFA10-2 program and logMAR VA and investigated the correlations among several factors related to the progression of RP.

## 2. Materials and Methods

We retrospectively studied the medical records of 922 patients with RP between 2009 and 2019 at Chiba University Hospital. We selected RP patients who underwent five or more VA tests and visual field tests involving at least one eye during a period of 5 years or more. Of the 922 patients, a total of 235 eyes from 121 patients were evaluated. The diagnosis of RP was based on the clinical history, funduscopic appearance, visual field test results, optical coherence tomography (OCT) findings, and full-field electroretinogram findings recorded according to the International Society for Clinical Electrophysiology of Vision standardized conditions. Patients with atypical RP, such as sectorial, central, secondary, or unilateral RP, were excluded from this study. Patients with other ocular diseases or disorders that affect visual function (for example, cystoid macular edema, macular hole, vitreo-macular traction, epiretinal membrane, advanced cataract, and advanced posterior capsular opacification) and eyes with a history of intraocular surgery, including cataract surgery during the study period, were excluded. We interviewed the patients and created detailed family trees for each to determine the pattern of inheritance. The patients were followed up once per year. At follow-up, patients routinely underwent visual automated static perimetry (HFA; Model 750; Carl Zeiss Meditec, Inc., Dublin, CA, USA) in addition to the measurement of best-corrected visual acuity (BCVA), slit lamp fundus examinations, intraocular pressure measurement, and spectral-domain OCT (SD-OCT; Heidelberg Engineering, Heidelberg, Germany). BCVA was examined with a standard Japanese decimal VA chart and system charts (SC-2000 Nidek Instruments, Gamagori, Japan) at 5 m and was converted to logMAR units. VA while counting fingers, hand motion, light perception, and no light perception were assigned logMAR values of 1.85, 2.3, 2.8, and 2.9, respectively [30] [31]. The HFA value was recorded on the same day as the other examinations, including the VA test, using the central 10-2 SITA-standard program. We excluded patients when the test reliability was not satisfactory with a HFA10-2 fixation loss score ≥ 20% or with either false-positive or false-negative errors ≥ 33%. We further investigated the average MD value of the central four points of the HFA10-2 numerical display as the S4. Since the decibel value is based on a logarithmic scale, we converted the value of each measured point in decibels to 1/Lambert (linear unit) and subsequently averaged the values when we calculated the average sensitivities of S4. Subsequently, we converted the value to dB.

Patients were classified into three groups: mild RP, eyes with the MD equal to or higher than -0.5 dB; moderate RP, eyes with the MD higher than -25.0 dB and lower than -0.5 dB; and late RP, including eyes with the MD equal to or lower than -25.0 dB. The values obtained from both the eyes were included in the model. The Kruskal–Wallis test and chi-square test were used to compare the three groups' differences in terms of the characteristics of the patient groups.

Linear mixed-effect models were used to determine the changes in the MD, sensitivity of S4, and VA (logMAR) with increasing time. The values obtained from both the eyes were included in the analysis. The dependent variables were the MD, S4, and VA, with time as a fixed effect and participants and eyes (left and right) as a random effect (intercept). In addition, to evaluate the effect of the baseline MD, sex, and hereditary form on the changes in the MD, S4, and VA over time, we added the fixed effects of factors (model 1, baseline MD group; model 2, sex; and model 3, hereditary form), and the interaction term between each factor and time to the linear mixed model is described above. The fixed effect was the time, and the random factors were the participants and eyes (intercept). In a simple regression analysis, we converted the MD values on a logarithmic scale to a linear scale (MD (1/Lambert)), to determine the percentage MD reduction rate. Subsequently, we constructed a linear mixed model with MD (1/Lambert) as an outcome. The yearly progression rate is represented as a decrease in the average initial MD (1/Lambert). Statistical significance was set at *p* < 0.05. All statistical analyses were performed using the SAS statistical software package (version 9.4; SAS Institute, Cary, USA).

## 3. Results

The demographic data of this study are shown in Table 1. The mean age at baseline was 52.5 (range: 10–81) years, and 55.3% were female participants. The mean follow-up year was 6.71. The hereditary forms were autosomal dominant (AD) in 13 cases, autosomal recessive (AR) in 13 cases, and sporadic in 95 cases. None of the patients had an X-linked RP. With respect to the baseline MD, the three groups were as follows: mild RP group, 60 eyes; moderate RP group, 138 eyes; and late RP group, 37 eyes. No significant differences in age, sex, or hereditary form distribution were found between the baseline MD groups.

Table 2 shows the 3 linear mixed models. All models include random intercepts for each subject over time. The coefficient of time (years) of each model is the fixed effect of the slopes or the average progression rate. The mean progression rate of the MD for all subjects was −0.37 dB/year (95% confidence interval (CI), −0.41 to −0.33; *p* < 0.001) or− 2.13% (95% CI, −2.81% to −1.44%; *p* < 0.001) on a linear scale (1/Lambert). The progression rate of sensitivity for the S4 was −0.25 dB/year (95% CI, −0.31 to −0.20; *p* < 0.001) and 0.018/year (95% CI, 0.015 to 0.020; *p* < 0.001) for VA.

Figure 1 shows the results of the analysis of the effects of variables on MD progression rates. A linear mixed model with an interaction term was used to determine the changes in the MD. All models included one of the variables (baseline MD, sex, and hereditary form), time (years), and an interaction between the variable and time, as well as random intercepts for time for each subject. The MD of the moderate RP group showed a faster decrease than that of the late RP group (difference: −0.22 dB/year, *p* < 0.001) and the mild RP group (difference: −0.29 dB/year, *p* < 0.001) (Figure 1). Sex did not show a statistically significant interaction between times on the MD progression rate. For hereditary form, the MD of the AD group showed a slower decrease than that of the sporadic group (difference: 0.14 dB/year, *p* = 0.02).

Figure 2 shows the results of the analysis of the effects of variables on S4 progression rates. The S4 progression rates of the late RP and moderate RP groups showed a faster decrease than those of the mild RP group (difference: late group, −0.24 dB/year, *p* = 0.011; moderate group, −0.30 dB/year, *p* < 0.001). The S4 of the female group had a slower decrease than that of the male group (difference: 0.13 dB/year, *p* = 0.024). The hereditary form did not show a statistically significant interaction between times on the S4 progression rate.

Figure 3 shows the results of the analysis of the effect of variables on logMAR VA progression rates. VA of the moderate and mild RP groups had a slower increase than that of the late group (difference: moderate group, −0.011/year, *p* = 0.0062; mild group, −0.017/year, *p* < 0.001). VA of females had a slower increase than that of males (difference: −0.015/year, *p* < 0.001). For hereditary forms, VA of the AD and AR groups had a slower increase than that of the sporadic group (difference: AD, −0.009/year, *p* = 0.034; AR, −0.010/year, *p* = 0.043).

Figure 4 shows the plots of the MD, S4, and logMAR VA for all patients in the mild, moderate, and late groups.

## 4. Discussion

We investigated the visual function changes in 235 eyes of 121 patients using data from the HFA10-2 program and a VA test for at least 5 years. We classified patients into three groups, mild RP, moderate RP, and late RP, to examine whether there is a difference in the natural course of central visual field sensitivity on the basis of the HFA perimeter and VA for each stage in this study. We further investigated whether sex and hereditary forms affect the progression rate. Although a few studies have shown the natural course of visual sensitivities using automated static perimetry [21, 32, 33], we included a large number of patients with a long observation period in this study.

Our result revealed that the mean reduction of the MD for all subjects was −0.37 dB/year (Table 2). Nakazawa et al. reported that progression rate of the mean MD for a period of 49.2 months for 14 control RP patients was -0.89 dB/year [7]. Fujiwara et al. reported that the mean MD slope of 118 RP patients was -0.47 dB/year [33]. The mean reduction of the sensitivity for S4 was −0.25 dB/year. Progression rate of the mean sensitivity for S4 of 45 patients was reported to be -0.33 dB/year in Sayo's study [21], -0.58 dB/year in Fujiwara's study, and -1.29 and -1.75 in the right and left eyes, respectively, in Nakazawa's study [32]. Overall, the progression rates of the HFA 10-2 values were reported to be faster in the previous reports than in our study. The presumed reason is the difference in the number of patients and observation period and the difference in the distribution of stages and study design. For example, patients whose baseline MD was less than -30 dB or more than -5 dB were excluded from Sayo's study.

The mean reduction in logMAR VA for all subjects in this study was 0.018 per year. Although there are very few reports on the natural course of VA in RP patients, Ogino et al. reported that the mean VA progression slope of 19 RP patients was 0.015 dB/year [20]. These results are similar to those of our study.

Few reports have investigated the progression rate of the MD as per the stage of RP. Sayo et al. reported that the mean baseline MD (-17.9 dB) was used to compare the progression of the two groups, and the MD progression rate was not significantly different between the two groups [21]. Fast progression in the moderate group (Figure 1) may be due to the changes in the MD value that were affected by the large number of measurement points in the HFA10-2 program. Moreover, progression of the mild group was underestimated because they have lost visual sensitivity mainly outside the central 10 degrees.

Our results showed that the S4 progression rates of the late RP and moderate RP groups showed a faster decrease than those of the mild RP group (Figure 2). In Sayo's study, progression was fast in the S4 in the advanced RP group (baseline MD < −17.9 dB) [21]. Ogino et al. reported that the participants with short ellipsoid zone (EZ) length as evaluated by OCT progressed faster in the central 4 points area than in other areas and those with long EZ length progressed faster in the peripheral area [20]. These results were consistent with our findings.

To the best of our knowledge, there have been no reports comparing the progression of VA with the stages of RP. Iijima reported a high correlation between VA and retinal sensitivity in the central 2 deg in the HFA 10-2 program. In contrast, Ogino et al. reported that VA and visual field were not related. The reason for the difference in these reports may be that VA is a test of the point function of the fovea, while the visual field test is an indicator of two-dimensional visual function.

Since the central visual function is mainly impaired in the terminal stage, while the peripheral vision is impaired in the earlier stage, our progression rate results for each stage of RP of the mean sensitivity for the S4 and logMAR VA are reasonable. These results indicated that the retinal sensitivity for the S4 and logMAR VA would be more appropriate than the MD values of the HFA10-2 program when assessing central vision function. Therefore, these two parameters may be suitable parameters for the assessment of the terminal stage.

Some studies revealed that the progression of visual sensitivities or the EZ length on OCT varied depending on the hereditary form [24–26]. However, several studies have reported that the differences among the hereditary forms were not significant [21, 33, 34]. Our results showed a significant difference between sporadic and AD groups for the MD and between sporadic and AD groups and sporadic and AR groups for VA. Jauregui et al. reported that the progression was slowest in the AD group [24], which is consistent with our results. However, genetic testing was not performed in our study, and the sample size was small; further research on the difference in the rate of progression of visual function in RP patients between the genotypes is needed.

Our study showed differences in the progression rates of the S4 and VA based on sex. The presence of estrogen receptors in different retinal layers has been reported [35]; moreover, biological sex and sex hormone profiles are considered an important cause of functional and structural differences in the retina [36]. Studies using mice have clarified the differences in retinal structure between males and females and found that retinal function, which was measured by multifocal electroretinography, is better in females of reproductive age than in males and older females [37]. Moreover, some studies have indicated that progestin therapy appears to improve the course of RP [27–29]. Several past studies have shown no difference in the progression rate of the MD, S4, and retinal structure according to sex [21, 25, 33]. These results, which are different from ours, could be due to the differences in sample size or selection bias. Our results indicate that there might be differences in the progression of central vision function according to sex.

In the analysis of MD progression rates over time, the baseline MD and hereditary form were found to be associated factors (Figure 1). As for the confounding factors, no statistically significant correlation was found in the association analysis of patient characteristics (Table 1); thus, we concluded that no confounding had occurred. In other words, the baseline MD and hereditary form were considered to have independent effects on the temporal changes in the MD. Similarly, for the analysis of S4 and VA progression rates (Figures 2 and 3), there was no confounding between the baseline MD, sex, and hereditary form (Table 1).

This study has several limitations. First, the number of participants was small. Therefore, it was difficult to perform a stratified analysis for each genetic form and sex with the number of cases. Second, selection bias was inevitable because only those who could test for the HFA10-2 program were enrolled, and a smaller number of patients were enrolled in the mild and late groups than in the moderate group. Third, genetic testing of the participants was not performed, although we interviewed them regarding their family history and created detailed family trees to determine the pattern of inheritance. The number of AD/AR cases in this study was smaller than those in previous reports [38, 39]. Since we inferred the genetic form from the pedigree, AD/AR cases might have been included within the sporadic cases. There were more AD, AR, and XL cases among the 922 participants identified during the medical record search; however, they were excluded from the study because they did not meet the inclusion criteria or fulfilled the exclusion criteria. The results of this study should be interpreted with caution since genetic testing was not performed. Further studies using genetic testing are needed. Fourth, we considered that it was inappropriate to use dB when we calculated the average of the central four points of the HFA10-2 program, as dB is a logarithmic scale. Thus, we converted the logarithmic scale (dB) to linear scale (1/Lambert) when calculating the central four points of the HFA10-2 program. However, the logarithmic scale (dB) is more familiar to the clinicians than the linear scale (1/Lambert); moreover, previous studies used a logarithmic scale when calculating the progression rate of the sensitivity of the HFA10-2 program [32, 33]; we selected the logarithmic scale, except for the calculation of the central four points and the year progression rate of the MD and S4 in the simple regression analysis. Liebmann et el. pointed out that the rate of progression is underestimated in early stages and overestimated in severe stages when measuring glaucoma progression on a logarithmic scale [40]. If we selected a linear scale (1/Lambert) in every other analysis, the results might be different. Fifth, we did not determine the onset of symptoms. The reason was that pathological findings occur before the onset of subjective symptoms, and the period from that point to the awareness of symptoms varies between patients. Moreover, the patients' memories regarding the onset of subjective symptoms were ambiguous, thus making it more difficult to determine the exact date of onset.

## 5. Conclusions

Our results revealed that the progression rates of VA and visual field tests differed as per the RP stage, and the appropriate tests for evaluation may differ depending on the stage of RP. Moreover, inheritance form and sex may affect the progression rate. Our results can be useful in predicting the natural course of patients with RP.

## Figures and Tables

**Figure 1:** Analysis of the effect of variables on MD progression rate. CI: confidence interval; RP: retinitis pigmentosa; AD: autosomal dominant; AR: autosomal recessive; MD: mean deviation of the Humphrey central 10-2 program.

**Figure 2:** Analysis of the effect of variables on S4 progression rate. CI: confidence interval; RP: retinitis pigmentosa; AD: autosomal dominant; AR: autosomal recessive; S4: average sensitivity of central four points of the Humphrey central 10-2 program.

**Figure 3:** Analysis of the effect of variables on logMAR VA progression rate. CI: confidence interval; RP: retinitis pigmentosa; AD: autosomal dominant; AR: autosomal recessive; logMAR VA: logarithm of the minimum angle of resolution visual acuity.

**Figure 4:** Plots of visual sensitivities and visual acuity during follow-up years in all patients. logMAR VA: logarithm of the minimum angle of resolution visual acuity; MD: mean deviation of the Humphrey central 10-2 program; S4: average sensitivity of central four points of the Humphrey central 10-2 program.

**Table 1:** Demographic data for the participants.

	All data		Mild RP		Moderate RP		Late RP		*p* value
	RE	LE	RE	LE	RE	LE	RE	LE	
Number	121	114	32	28	69	69	20	17	
Age (years)	52.5 ± 16.2 (10 to 81)		52.8 ± 12.5 (10 to 76)		51.5 ± 16.7 (19 to 81)		55.5 ± 12.5 (21 to 78)		0.71
Sex (female %)	67 (55.3)		17 (53)		40 (57)		10 (50)		0.78
AD/AR/sporadic	13/13/95		4/2/26		8/8/53		1/3/16		0.77
Follow-up years	6.71 ± 1.7 (5-11)		6.96 ± 1.95 (5 to 11)		6.69 ± 1.7 (5 to 11)		6.35 ± 0.9 (5 to 8)		0.76
logMAR VA	0.17 ± 0.3 (-0.07 to 2)		0.05 ± 0.2 (-0.07 to 0.69)		0.15 ± 0.2 (-0.08 to 1)		0.48 ± 0.2 (-0.07 to 2)		<0.0001
MD (dB)	−13.52 ± 9.0 (-33.5 to 0.76)		−2.9 ± 1.6 (-4.9 to 0.76)		−14.2 ± 5.0 (-24.5 to 5.4)		−28.5 ± 2.8 (-33.5 to -25.1)		<0.0001
S4 (dB)	28.4 ± 6.5 (0.83 to 36.5)		32.6 ± 2.0 (27.8 to 36.5)		28.7 ± 4.5 (9.1 to 34.8)		20.2 ± 9.5 (0.83-32.8)		<0.0001

RE: right eye; LE: left eye; RP: retinitis pigmentosa; AD: autosomal dominant; AR: autosomal recessive; logMAR VA: logarithm of the minimum angle of resolution visual acuity; MD: mean deviation of the Humphrey central 10-2 program; S4: average sensitivity of central four points of the Humphrey central 10-2 program. Values are presented as mean ± standard deviation (range).

**Table 2:** Mean progression rate of MD, S4, and logMAR VA.

Outcome	Coefficient	95% CI	*p* value
MD (dB)			
Intercept	-11.89	-13.61, -10.18	<0.001
Time (years)	-0.37	-0.41, -0.33	<0.001
S4 (dB)			
Intercept	29.82	28.60, 31.04	<0.001
Time (years)	-0.25	-0.31, -0.20	<0.001
logMAR VA			
Intercept	0.113	0.051, 0.175	<0.001
Time (years)	0.018	0.015, 0.020	<0.001

CI: confidence interval; logMAR VA: logarithm of the minimum angle of resolution visual acuity; MD: mean deviation of the Humphrey central 10-2 program; S4: average sensitivity of central four points of the Humphrey central 10-2 program.

## Data Availability

All the data supporting our findings are contained within the manuscript.

## References

[1] Berson E. L., Sandberg M. A., Rosner B., Birch D. G., Hanson A. H. (1985). Natural course of retinitis pigmentosa over a three-year interval. *American Journal of Ophthalmology*.

[2] Berson E. L., Rosner B., Sandberg M. A. (1993). A randomized trial of vitamin A and vitamin E supplementation for retinitis pigmentosa. *Archives of Ophthalmology*.

[3] Berson E. L., Rosner B., Sandberg M. A. (2010). Clinical trial of lutein in patients with retinitis pigmentosa receiving vitamin A. *Archives of Ophthalmology*.

[4] Hoffman D. R., Hughbanks-Wheaton D. K., Spencer R. (2015). Docosahexaenoic acid slows visual field progression in X-linked retinitis pigmentosa: ancillary outcomes of the DHAX trial. *Investigative Ophthalmology & Visual Science*.

[5] Merin S., Obolensky A., Farber M. D., Chowers I. (2008). A pilot study of topical treatment with an alpha2-agonist in patients with retinal dystrophies. *Journal of Ocular Pharmacology and Therapeutics*.

[6] Bahrami H., Melia M., Dagnelie G. (2006). Lutein supplementation in retinitis pigmentosa: PC-based vision assessment in a randomized double-masked placebo-controlled clinical trial [NCT00029289]. *BMC Ophthalmology*.

[7] Nakazawa M., Ohguro H., Takeuchi K., Miyagawa Y., Ito T., Metoki T. (2011). Effect of nilvadipine on central visual field in retinitis pigmentosa: a 30-month clinical trial. *Ophthalmologica*.

[8] Vingolo E. M., Rocco M., Grenga P., Salvatore S., Pelaia P. (2007). Slowing the degenerative process, long lasting effect of hyperbaric oxygen therapy in retinitis pigmentosa. *Graefe’s Archive for Clinical and Experimental Ophthalmology*.

[9] Cehajic-Kapetanovic J., Xue K., Martinez-Fernandez de la Camara C. (2020). Initial results from a first-in-human gene therapy trial on X-linked retinitis pigmentosa caused by mutations in RPGR. *Nature Medicine*.

[10] Liu Y., Chen S. J., Li S. Y. (2017). Long-term safety of human retinal progenitor cell transplantation in retinitis pigmentosa patients. *Stem Cell Research & Therapy*.

[11] Busskamp V., Picaud S., Sahel J. A., Roska B. (2012). Optogenetic therapy for retinitis pigmentosa. *Gene Therapy*.

[12] da Cruz L., Dorn J. D., Humayun M. S. (2016). Five-year safety and performance results from the Argus II retinal prosthesis system clinical trial. *Ophthalmology*.

[13] Miura G., Sugawara T., Kawasaki Y. (2019). Clinical trial to evaluate safety and efficacy of transdermal electrical stimulation on visual functions of patients with retinitis pigmentosa. *Scientific Reports*.

[14] Holopigian K., Greenstein V., Seiple W., Carr R. E. (1996). Rates of change differ among measures of visual function in patients with retinitis pigmentosa. *Ophthalmology*.

[15] Grover S., Fishman G. A., Anderson R. J., Alexander K. R., Derlacki D. J. (1997). Rate of visual field loss in retinitis pigmentosa. *Ophthalmology*.

[16] Nowomiejska K., Brzozowska A., Koss M. J. (2016). Quantification of the visual field loss in retinitis pigmentosa using semi-automated kinetic perimetry. *Current Eye Research*.

[17] Grover S., Fishman G. A., Brown J. (1998). Patterns of visual field progression in patients with retinitis pigmentosa. *Ophthalmology*.

[18] Hirakawa H., Iijima H., Gohdo T., Imai M., Tsukahara S. (1999). Progression of defects in the central 10-degree visual field of patients with retinitis pigmentosa and choroideremia. *American Journal of Ophthalmology*.

[19] Iijima H. (2013). Visual loss and perimetric sensitivity in eyes with retinitis pigmentosa. *Japanese Journal of Ophthalmology*.

[20] Ogino K., Otani A., Oishi A., Kurimoto M., Sekiya T., Yoshimura N. (2013). Concentric division of 10° visual field tests in retinitis pigmentosa. *Japanese Journal of Ophthalmology*.

[21] Sayo A., Ueno S., Kominami T. (2017). Longitudinal study of visual field changes determined by Humphrey field analyzer 10-2 in patients with retinitis pigmentosa. *Scientific Reports*.

[22] Iijima H. (2012). Correlation between visual sensitivity loss and years affected for eyes with retinitis pigmentosa. *Japanese Journal of Ophthalmology*.

[23] Szlyk J. P., Fishman G. A., Alexander K. R., Revelins B. I., Derlacki D. J., Anderson R. J. (1997). Relationship between difficulty in performing daily activities and clinical measures of visual function in patients with retinitis pigmentosa. *Archives of Ophthalmology*.

[24] Jauregui R., Takahashi V. K. L., Park K. S. (2019). Multimodal structural disease progression of retinitis pigmentosa according to mode of inheritance. *Scientific Reports*.

[25] Sujirakul T., Lin M. K., Duong J., Wei Y., Lopez-Pintado S., Tsang S. H. (2015). Multimodal imaging of central retinal disease progression in a 2-year mean follow-up of retinitis pigmentosa. *American Journal of Ophthalmology*.

[26] Birch D. G., Locke K. G., Wen Y., Locke K. I., Hoffman D. R., Hood D. C. (2013). Spectral-domain optical coherence tomography measures of outer segment layer progression in patients with X-linked retinitis pigmentosa. *JAMA Ophthalmology*.

[27] Sánchez-Vallejo V., Benlloch-Navarro S., López-Pedrajas R., Romero F. J., Miranda M. (2015). Neuroprotective actions of progesterone in an in vivo model of retinitis pigmentosa. *Pharmacological Research*.

[28] Doonan F., O'Driscoll C., Kenna P., Cotter T. G. (2011). Enhancing survival of photoreceptor cells in vivo using the synthetic progestin Norgestrel. *Journal of Neurochemistry*.

[29] Doonan F., Cotter T. G. (2012). Norgestrel may be a potential therapy for retinal degenerations. *Expert Opinion on Investigational Drugs*.

[30] Grover S., Fishman G. A., Anderson R. J. (1999). Visual acuity impairment in patients with retinitis pigmentosa at age 45 years or older. *Ophthalmology*.

[31] Schulze-Bonsel K., Feltgen N., Burau H., Hansen L., Bach M. (2006). Visual acuities “hand motion” and “counting fingers” can be quantified with the Freiburg visual acuity test. *Investigative Ophthalmology & Visual Science*.

[32] Nakazawa M., Suzuki Y., Ito T., Metoki T., Kudo T., Ohguro H. (2013). Long-term effects of nilvadipine against progression of the central visual field defect in retinitis pigmentosa: an extended study. *BioMed Research International*.

[33] Fujiwara K., Ikeda Y., Murakami Y. (2018). Assessment of central visual function in patients with retinitis pigmentosa. *Scientific Reports*.

[34] Xu M., Zhai Y., MacDonald I. M. (2020). Visual field progression in retinitis pigmentosa. *Investigative Ophthalmology & Visual Science*.

[35] Kobayashi K., Kobayashi H., Ueda M., Honda Y. (1998). Estrogen receptor expression in bovine and rat retinas. *Investigative Ophthalmology & Visual Science*.

[36] Yamashita H., Sugihara K., Yamada C., Tsutsumi S., Iwaki Y. (2010). Effect of estrogen on electroretinographic responses in streptozotocin-induced diabetic female rats. *Experimental Eye Research*.

[37] Chaychi S., Polosa A., Lachapelle P. (2015). Differences in retinal structure and function between aging male and female Sprague-Dawley rats are strongly influenced by the estrus cycle. *PLoS One*.

[38] Hayakawa M., Matsumura M., Ohba N. (1993). A multicenter study of typical retinitis pigmentosa in Japan. *Japanese Journal of Ophthalmology*.

[39] Hayakawa M., Fujiki K., Kanai A. (1997). Multicenter genetic study of retinitis pigmentosa in Japan: I. Genetic heterogeneity in typical retinitis pigmentosa. *Japanese Journal of Ophthalmology*.

[40] Liebmann K., De Moraes C. G., Liebmann J. M. (2017). Measuring rates of visual field progression in linear versus nonlinear scales: implications for understanding the relationship between baseline damage and target rates of glaucoma progression. *Journal of Glaucoma*.

